RETRACTED

# Establishment of a Nomogram Model for Predicting Cardiovascular and Cerebrovascular Events in Diabetic Nephropathy Patients Receiving Maintenance Hemodialysis

**DOI:** 10.1155/2022/2909726

**Published:** 2022-07-07

**Authors:** Xiaobing Liu, Caili Yan, Xiuxiu Niu, Jiechun Zeng

**Affiliations:** ^1^Department of Endocrinology, Huidong People's Hospital, Huizhou, China; ^2^Infection Management Department, Huizhou First Hospital, Huizhou, China; ^3^Department of Science and Education, Huidong People's Hospital, Huizhou, China

## Abstract

**Objective:**

The objective of this study is to explore the risk factors of cardiovascular and cerebrovascular events (CCE) in patients with diabetic nephropathy (DN) receiving maintenance hemodialysis, and to establish a nomogram model on this basis.

**Method:**

144 patients with DN receiving maintenance hemodialysis from February 2020 to February 2021 were selected and followed up for 12 months. They were divided into the occurrence and nonoccurrence groups according to whether CCE occurred. The multivariate logistic regression analysis was used to analyze the influencing factors of CCE, and a predictive nomogram model was established. The receiver operating characteristic (ROC) curve was drawn to evaluate the predictive effect of the nomogram model. The Hosmer-Lemeshow method was used to test the calibration degree.

**Results:**

Among the patients, 63 patients (43.75%) encountered CCE. Multivariate logistic regression analysis showed that age >60 years old, history of CCE, dialysis age >12 months, systolic blood pressure >140 mmHg, blood phosphorus level >1.5 mmol/L, triglyceride (TG) level >2.30 mmol/l, adiponectin (ADPN) level <5 mg/L, high-sensitivity-C-reactive protein (hs-CRP) level >10 mg/L, hemoglobin (Hb) level <120 g/L, serum creatinine (SCr) level >720 *μ*mol/L, and albumin (ALB) level <40 g/L were independent risk factors for CCE. Based on the above independent risk factors, a nomogram model of CCE was created. ROC curve analysis showed that the area under curve for predicting CCE was 0.881 (95% CI: 0.833~0.919), indicating that the nomogram model had great predictive effect. The Hosmer-Lemeshow method showed that the calibration curve was in good agreement with the standard curve.

**Conclusion:**

Age, history of CCE, dialysis age, systolic blood pressure and serum phosphorus, and TG, ADPN, hs-CRP, Hb, SCr, and ALB levels are all influencing factors for the occurrence of CCE in patients with DN receiving maintenance hemodialysis, and the nomogram model has a great predictive effect on CCE.

## 1. Introduction

Diabetic nephropathy (DN) is a common microvascular complication of diabetes, with its incidence increasing in recent years. It has various clinical manifestations, mainly including edema, proteinuria, and hypertension, and may result in renal failure in severe cases, which is one of the main causes of end-stage renal disease, seriously threatening the lives of patients [1, 2]. At present, maintenance hemodialysis is a major method for the treatment of DN, which plays the role of the kidneys in purifying the blood and is of great significance to patients by saving their lives [3]. However, long-term hemodialysis damages vascular endothelial function, leads to atherosclerosis and other problems, and increases the risk of cardiovascular and cerebrovascular events in patients [4]. A previous study [5] pointed out that DN patients might encounter various cardiovascular and cerebrovascular events such as heart failure, myocardial infarction, and cerebral infarction during maintenance hemodialysis, increasing the risk of death. Therefore, it is necessary to assess the risk of cardiovascular and cerebrovascular events in DN patients receiving maintenance hemodialysis as soon as possible and establish an effective predictive model to provide guidance on clinical treatment and improve prognoses.

RETRACTED

A nomogram model is satisfactorily accurate, visual, and easy to understand and can be used to predict disease outcomes [6]. A related study reported [7] that the nomogram prediction model could be used for risk monitoring and prevention of patients with diabetic foot ulcers. Li et al. [8] showed that the nomogram model predicted the probability of withdrawal in peritoneal dialysis patients. In addition, You et al. [9] developed a simple and practical nomogram prediction model that could assess the risk of cardiovascular events in long-term hemodialysis patients with chronic kidney disease. However, there is no accurate nomogram model to assess the risk factors for cardiovascular events in DN patients receiving maintenance hemodialysis. Therefore, in this study, the clinical data of the selected patients with DN receiving maintenance hemodialysis were evaluated, and a nomogram prediction model for the risk of cardiovascular and cerebrovascular events was created to provide a reference for clinical assessment and treatment, as reported below.

## 2. Methods

### 2.1. General Data

Based on the approval from the Ethics Committee of Huidong People's Hospital (2022-034), 144 patients with DN receiving maintenance hemodialysis, who have been admitted to the hospital during the period from February 2020 to February 2021, were selected.

Inclusion criteria are as follows: patients who ① met the relevant criteria specified in *Diagnosis and Treatment of Diabetic Nephropathy* [10], and were diagnosed with DN; ② had end-stage diabetic nephropathy and were receiving maintenance hemodialysis in the hospital; ③ had a dialysis age that was more than 3 months; ④ have no intellectual and consciousness impairment and can answer the doctor's questions independently and clearly; and ⑤ signed the informed consent for this study.

RETRACTED

Exclusion criteria are as follows: ① renal transplant recipients; ② patients with severe infection, peritoneal dialysis or malignant tumor, liver and lung and other serious chronic diseases; ③ complicated with respiratory failure or basic diseases of the nervous system; ④ pregnant or lactating; and ⑤ patients with infectious diseases and mental history.

Elimination criteria are as follows: ① patients who lost to follow-up and ② patients who died due to other diseases or accidents.

### 2.2. Dialysis Method

All patients were treated with 4008 s dialysis machines (Fresenius Group, Germany) and disposable polysulfone membrane dialyzers for maintenance hemodialysis. They received dialysis three times a week, with a period of 4-4.5 h each time. An autologous arteriovenous fistula or a semi-permanent central venous catheter was used as vascular access. Dialysis was performed with standard bicarbonate dialysate (Sangon Biotech (Shanghai) Co., Ltd.) at a blood flow velocity of 200-250 ml/min, a dialysate K^+^ concentration of 2.00 mmol/L and a Ca^2+^ concentration of 1.50 mmol/L, and a speed of 500 ml/min, and low-molecular-weight heparin calcium injection and heparin sodium injection were used for anticoagulation. All patients were monitored in real time during treatment and given other basic treatments, such as correction of anemia, control of blood pressure, and correction of calcium-phosphorus metabolism disorder.

### 2.3. Observation Indicators

Clinical data were collected on admission, including gender, age, body mass index (BMI), diabetes duration, diabetic nephropathy duration, smoking history, history of cardiovascular and cerebrovascular diseases, blood pressure, and dialysis age.

When the patients were enrolled and every 3 months after enrollment, the laboratory indexes were examined. Fasting veins were collected from all patients before dialysis. After each patient got up in the morning and rested for 15 minutes, they continuously measured the upper limb arterial blood pressure three times with an electronic sphygmomanometer (purchased from Omron medical (China) Co., Ltd.). Systolic and diastolic blood pressure was recorded before dialysis, and peripheral venous blood was collected. Then, the blood samples were separated, and the levels of blood triglyceride (TG), serum phosphorus, serum adiponectin (ADPN), high-sensitivity C-reactive protein (hs-CRP), hemoglobin (HB), serum creatinine (SCR), and serum albumin (ALB) were detected by enzyme-linked immunosorbent assay (ELISA, Nanjing Weideng Medical Co., Ltd., China) and automatic biochemical analyzer.

RETRACTED

### 2.4. Outcome

We included cardiovascular and cerebrovascular events after hemodialysis as a result. Cardiovascular and cerebrovascular end points in DN patients included myocardial infarction, heart failure, malignant arrhythmia, ischemic heart disease, sudden death, and cerebral infarction. Patients with cardiovascular and cerebrovascular events were divided into occurrence groups, and other patients were divided into nonoccurrence groups.

### 2.5. Statistical Analysis

The SPSS26.0 software was used for statistical analysis. The measurement data was described with mean ± standard deviation (SD) and tested with Student's t-test. And the count data was described with “%” and compared with *χ*^2^ test. Multivariate logistic regression analysis was used to analyze the risk factors for cardiovascular and cerebrovascular events in DN patients receiving maintenance hemodialysis. A nomogram model was created based on the risk factors, and the receiver operating characteristic (ROC) curve was used to assess the effectiveness of the nomogram model in predicting cardiovascular and cerebrovascular events in diabetic nephropathy patients receiving maintenance hemodialysis. If *P* < 0.05, the difference was statistically significant. The Hosmer-Lemeshow method was used to test the predictive effect of the nomogram model; when *P* > 0.05, it indicated a great degree of calibration.

## 3. Results

### 3.1. Basic Characteristics of Patients

Among the 144 patients with DN receiving maintenance hemodialysis enrolled in this study, these patients were aged 50-72, with an average age of 60.48 ± 10.06; their BMI was within a range of 18.45-28.12 kg/m^2^, with an average of 23.27 ± 2.06 kg/m^2^; their courses of diabetes ranged from 1 year to 9 years, with an average of 60.41 ± 10.04 months; their courses of diabetic nephropathy ranged from 9 months to 6 years, with an average of 50.06 ± 8.35 months; and their dialysis ages ranged from 6 months to 4 years, with an average of 26.32 ± 4.34 months.

And 63 patients encountered cardiovascular and cerebrovascular events during the 12-month follow-up period, with an incidence of 43.75% (63/144). There was no statistically significant difference in gender, BMI, course of diabetes, course of diabetic nephropathy, smoking history, and diastolic blood pressure between the occurrence group and the nonoccurrence group (*P* > 0.05). The constituent ratios of patients who had a history of cardiovascular and cerebrovascular diseases, a dialysis age >12 months, and a serum adiponectin (ADPN) level <5 mg/L in the occurrence group were higher than those in the nonoccurrence group (*P* < 0.05), and the ages and hs-CRP, systolic blood pressure, blood phosphorus, TG, and SCr levels of the patients in the occurrence group were higher than those in the nonoccurrence group (*P* < 0.05); the Hb and ALB levels of the patients in the occurrence group were lower than those in the non-occurrence group (*P* < 0.05) (see Table 1 for details).

RETRACTED

### 3.2. Multivariate Analysis of Cardiovascular and Cerebrovascular Events

Multivariate logistic regression analysis showed that age >60 years old, history of cardiovascular and cerebrovascular diseases, dialysis age >12 months, systolic blood pressure >140 mmHg, blood phosphorus level >1.5 mmol/L, TG level >2.30 mmol/l, ADPN level <5 mg/L, hs-CRP level >10 mg/L, Hb level <120 g/L, SCr level >720 *μ*mol/L, and ALB level <40 g/L were independent risk factors for cardiovascular and cerebrovascular events in patients with DN receiving maintenance hemodialysis (*P* < 0.05) (see Table 2 for details).

### 3.3. Creation and Validation of a Nomogram Model and Its Predictive Effect

A nomogram model for predicting the risk of cardiovascular and cerebrovascular events in patients is created with the 11 independent risk factors screened by multivariate logistic regression analysis as predictors, as shown in Figure 1. ROC curve analysis showed that the area under curve (AUC) for predicting cardiovascular and cerebrovascular events in patients was 0.881 (95% CI: 0.833~0.919), the sensitivity was 69.32% and the specificity was 87.92%, indicating that the nomogram model had a great predictive effect (Figure 2). The Hosmer-Lemeshow test method is used to test the predictive effect of the nomogram model (*χ*^2^ = 6.472, *P* = 0.215), and it is found that the calibration curve was in good agreement with the standard curve, as shown in Figure 3.

## 4. Discussion

DN is caused by long-term abnormal glucose metabolism, which results in decreased glomerular filtration rate and glomerular sclerosis, and thus leads to damage to renal functions, causing great harm to the health of patients [11]. At present, maintenance hemodialysis can be used to effectively prolong the survival time of patients; however, long-term hemodialysis leads to the occurrence of cardiovascular and cerebrovascular events and increases the risk of death [12]. In this study, the incidence of cardiovascular and cerebrovascular events in 144 patients with DN receiving maintenance hemodialysis was 43.75%, which is basically consistent with the results of Mei et al. [13] and Luo et al. [14]. It shows that the risk of cardiovascular and cerebrovascular events in patients with diabetic nephropathy receiving maintenance hemodialysis is relatively high. Therefore, it is necessary to analyze the influencing factors of cardiovascular and cerebrovascular events in maintenance hemodialysis patients with diabetic nephropathy, so as to provide guidance for intervention and management of high-risk patients in clinical practice.

RETRACTED

In this study, it was found through logistic regression analysis that age, history of cardiovascular and cerebrovascular diseases, dialysis age, systolic blood pressure and serum phosphorus, and TG, ADPN, hs-CRP, Hb, SCr, and ALB levels are all influencing factors of the occurrence of cardiovascular and cerebrovascular events in diabetic nephropathy patients receiving maintenance hemodialysis. With the increase in age, patients experience a decline in bodily functions and a decrease in the elasticity of arterial vascular walls and often suffer from various underlying diseases, so their tolerance to maintenance hemodialysis decreases, and the probability of the occurrence of cardiovascular and cerebrovascular events increases. With the increase in dialysis age, the retention of toxins caused by the disease, the increase in volume load, and the hemodynamic changes during dialysis have adverse effects on the cardiac functions of the patients, leading to the gradual deterioration of their cardiac functions. As the dialysis age increases, the risk of developing dialysis-related amyloidosis increases, and the risk of the occurrence of cardiovascular and cerebrovascular events increases accordingly. When patients had a history of cardiovascular and cerebrovascular diseases, they might suffer cardiovascular and cerebrovascular damage, so the probability of cardiovascular and cerebrovascular adverse events was higher, which was consistent with relevant reports [13]. Hypertension can cause damage to vascular endothelial cells, accelerate coronary atherosclerosis, block coronary arteries, and lead to cardiovascular and cerebrovascular accidents. It was found in a related survey [15] that an increase of 10 mmHg in systolic blood pressure increased the risk of coronary heart disease by approximately 20%. When the blood phosphorus level stays high for a long period, calcification of blood vessels and heart valves might be caused, which promotes the secretion of myocardial injury markers, leading to apoptosis of myocardial cells and myocardial damage and increasing the risk of cardiovascular and cerebrovascular events [16]. TG is one of the important components that cause atherosclerosis. Excessive TG content increases blood viscosity, decreases blood flow velocity, and accelerates blockage of blood vessels, causing cardiovascular and cerebrovascular diseases [17]. As an endogenous protein secreted by adipocytes, ADPN can protect vascular endothelial function and resist atherosclerosis. When the ADPN level is significantly reduced, its functions of protecting vascular endothelium and resisting atherosclerosis decline. A previous study [18] showed that the serum ADPN levels in patients with chronic kidney disease were closely related to the risk of adverse cardiovascular outcomes before dialysis, and could promote the progression of coronary calcification and increase the risk of cardiovascular events, which were similar to the results of this study. hs-CRP is an indicator that reflects the body's inflammatory response, and high expression of hs-CRP can aggravate the damage to vascular endothelial cells and increase the risk of death. A study [19] showed that hs-CRP is a risk factor for adverse cardiovascular events in patients receiving hemodialysis, which is consistent with the results of this study. In addition, ALB and Hb play a significant role in maintaining the normal metabolism of the body. Low ALB and Hb levels often indicate poor nutritional status of the body. After receiving maintenance hemodialysis, patients suffer increased malnutrition, leading to the occurrence of anemia, which can increase the cardiac load and stroke volume, cause myocardial hypoxia and thus lead to myocardial damage, and may also lead to water-sodium retention and thus lead to ventricular dilatation, thereby increasing the risk of cardiovascular and cerebrovascular events [20]. After glomerular filtration, SCr is excreted. When a patient's renal function is impaired, SCr cannot be cleaned up in time, leading to its accumulation in the body, which results in metabolic disorder, increases the burden on the kidneys, and tends to cause cardiovascular and cerebrovascular diseases [21]. Zhang et al. [22] pointed out that SCr is a risk factor for cardiovascular events in chronic kidney disease patients receiving maintenance hemodialysis, which further indicates that SCr is associated with cardiovascular and cerebrovascular events in patients receiving maintenance hemodialysis. The occurrence of cardiovascular and cerebrovascular events is the result caused by a variety of factors, and the above indicators have certain value in predicting cardiovascular and cerebrovascular events in diabetic nephropathy patients receiving maintenance hemodialysis.

RETRACTED

A nomogram model draws multiple predictors on one plane based on multifactor regression analysis and can get the predicted probability of each individual's outcome according to the corresponding algorithm, which is highly operable and accurate [23]. In this study, 11 independent risk factors screened by multivariate logistic regression analysis were used as predictors to create a nomogram model for predicting the risk of cardiovascular and cerebrovascular events in diabetic nephropathy patients receiving maintenance hemodialysis. It was found through internal and external validations that the nomogram model has great specificity and sensitivity and can properly predict the risk of cardiovascular and cerebrovascular events in diabetic nephropathy patients receiving maintenance hemodialysis. The prediction result is consistent with the actual risk of cardiovascular and cerebrovascular events, indicating that the model has great accuracy and thus has great value in clinical practice. Clinicians can predict the possibility of cardiovascular and cerebrovascular events in diabetic nephropathy patients receiving maintenance hemodialysis based on the nomogram model and take preventive measures in advance to minimize the occurrence of cardiovascular and cerebrovascular events in diabetic nephropathy patients receiving maintenance hemodialysis.

To sum up, age, history of cardiovascular and cerebrovascular diseases, dialysis age, systolic blood pressure and serum phosphorus, and TG, ADPN, hs-CRP, Hb, SCr, and ALB levels are all influencing factors of the occurrence of cardiovascular and cerebrovascular events in diabetic nephropathy patients receiving maintenance hemodialysis, and the nomogram model created on this basis has a great predictive effect on cardiovascular and cerebrovascular events in diabetic nephropathy patients receiving maintenance hemodialysis, which can provide significant guidance in clinical practice.

## Figures and Tables

**Figure 1:** Nomogram model for predicting the risk of cardiovascular and cerebrovascular events in diabetic nephropathy patients receiving maintenance hemodialysis.

**Figure 2:** ROC curve for prediction of cardiovascular and cerebrovascular events in diabetic nephropathy patients receiving maintenance hemodialysis with the nomogram model.

**Figure 3:** Calibration curve graph for prediction with the nomogram model.

**Table 1:** Comparison of clinical data between the occurrence group and the nonoccurrence group.

Clinical data	Occurrence group (*n* = 63)	Nonoccurrence group (*n* = 81)	*t*/*χ*^2^ value	*P* value
Gender (%)				
Male	36 (57.14)	51 (62.96)	0.502	0.479
Female	27 (42.86)	30 (37.04)		
Age (years old)	63.66 ± 11.14	58.01 ± 10.24	3.160	0.002
BMI (kg/m^2^)	23.45 ± 2.16	23.13 ± 2.04	0.910	0.364
Course of diabetes	59.32 ± 8.16	61.25 ± 9.03	1.327	0.187
Course of diabetic nephropathy (months)	49.62 ± 7.46	50.41 ± 8.25	0.594	0.553
History of cardiovascular and cerebrovascular diseases				
Yes	35 (55.56)	31 (38.27)	4.264	0.039
No	28 (44.44)	50 (61.73)		
Smoking history				
Yes	33 (52.38)	49 (60.49)	0.951	0.329
No	30 (47.62)	32 (39.51)		
Systolic blood pressure (mmHg)	146.14 ± 18.17	137.42 ± 17.25	2.940	0.004
Diastolic blood pressure (mmHg)	85.14 ± 12.95	87.36 ± 12.61	1.036	0.302
Dialysis age (months)				
≤12	15 (23.81)	50 (61.73)	20.576	<0.001
>12	48 (76.19)	31 (38.27)		
Serum phosphorus (mmol/L)	1.66 ± 0.40	1.52 ± 0.34	2.268	0.025
TG (mmol/L)	2.42 ± 0.44	2.24 ± 0.41	2.531	0.012
ADPN (mg/L)				
≥5	27 (42.86)	51 (62.96)	5.770	0.016
<5	36 (57.14)	30 (37.04)		
hs-CRP (mg/L)	15.76 ± 3.12	7.42 ± 1.45	21.297	<0.001
Hb (g/L)	105.14 ± 15.92	122.35 ± 18.36	5.909	<0.001
SCr (*μ*mol/L)	825.14 ± 106.10	642.23 ± 88.17	11.294	<0.001
ALB (g/L)	36.24 ± 7.02	40.05 ± 7.64	3.075	0.003

RETRACTED

**Table 2:** Multivariate logistic regression analysis.

Influencing factor	*β* value	*SE*	*Waldχ* ^2^	*P* value	*OR* value	95% CI
Age >60 years old	1.359	0.399	11.601	<0.001	3.892	2.099~4.128
History of cardiovascular and cerebrovascular diseases	1.113	0.379	8.624	0.021	3.043	2.156~5.690
Dialysis age >12 months	1.572	0.435	13.060	<0.001	4.816	3.001~5.532
Systolic blood pressure >140 mmHg	1.306	0.453	8.312	0.001	3.691	3.658~6.524
Serum phosphorus >1.50 mmol/L	1.146	0.375	9.339	0.013	3.146	3.021~5.124
TG >2.30 mmol/L	1.246	0.436	8.167	0.004	3.476	3.218~5.159
ADPN <5 mg/L	1.554	0.467	11.073	0.007	4.730	4.239~6.408
hs-CRP >10 mg/L	1.674	0.463	13.072	<0.001	5.333	3.282~5.631
Hb <120 g/L	1.507	0.527	8.177	<0.001	4.513	4.429~7.556
SCr >720 *μ*mol/L	1.598	0.585	7.462	<0.001	4.943	4.352~6.769
ALB <40 g/L	1.341	0.504	7.079	0.001	3.823	3.208~5.495

## Data Availability

The data used to support the findings of this study are available from the corresponding author upon request.
